The article "The Expression of the Long Noncoding RNA AFAP1-AS1 in Laryngeal Carcinoma Affects the Proliferation, Invasion, Migration, and Apoptosis of TU212 Cell Line" was retracted in 2023. Reasons: unreliable results or conclusions; lack of ethics approval or compliance; concerns about the data; concerns about the peer review.

# The Expression of the Long Noncoding RNA AFAP1-AS1 in Laryngeal Carcinoma Affects the Proliferation, Invasion, Migration, and Apoptosis of TU212 Cell Line

**DOI:** 10.1155/2022/2337447

**Published:** 2022-08-04

**Authors:** Xin Chen, Ziwei Hu, Liao Bing, Xinhua Zhu, Ke Liu, Yuehui Liu, Jianguo Liu

**Affiliations:** ^1^Otolaryngology Department of Youxian People's Hospital of Hunan Province, China; ^2^Department of Otolaryngology and Head and Neck Surgery, Guangzhou Red Cross Hospital Affiliated to Jinan University, China; ^3^Otolaryngology Head and Neck Surgery, Second Affiliated Hospital of Nanchang University, China

## Abstract

**Background:**

lncRNA AFAP1-AS1 has been linked to the pathogenesis of a wide range of tumors. Nevertheless, whether it plays a role in laryngeal carcinoma (LC) remains unclear.

**Methods:**

Twenty-nine pairs of LC and related normal tissues were collected for the detection of lncRNA AFAP1-AS1 using qRT-PCR. Correlation of lncRNA AFAP1-AS1 level and clinicopathological characters was assessed by the chi-square test. Impacts of lncRNA AFAP1-AS1 silencing on LC phenotypes were tested *in vitro* via CCK-8, clone formation, EdU staining, wound healing, flow cytometry, and Transwell assay.

**Results:**

Herein, a remarkable elevation of lncRNA AFAP1-AS1 was observed in LC patients. And higher lncRNA AFAP1-AS1 level was correlated to worse clinical pathological characteristics. Moreover, lncRNA AFAP1-AS1 silencing was revealed to repress TU212 malignant phenotypes.

**Conclusion:**

Our data suggested that lncRNA AFAP1-AS1 acts as an oncogene of LC *in vitro*.

## 1. Background

Laryngeal cancer (LC) is a malignant tumor in otolaryngology, among which 96%-98% consists of squamous cell carcinoma [1]. In comparison, others such as adenocarcinoma, basal cell carcinoma, poorly differentiated carcinoma, lymphosarcoma, and malignant lymphoma are rare [1]. Global cancer analysis data show that in 2002, there were 159,000 new cases and 90,000 deaths [2]. Cancer accounts for 2.4% of all male diseases and is 7-9 times more common in men than in women [1, 2]. In recent decades, the incidence of LC has increased significantly, and the onset age is mainly between 40 and 60 years. Although great progress has been made in the clinical treatment of LC in the past decades, including surgical intervention, radiotherapy, and chemotherapy, the prognosis of advanced LC patients remains unsatisfactory [3]. Therefore, exploring the molecular mechanisms underlying the carcinogenesis or progression of LC is crucial for the development of more effective therapeutic targets.

Long noncoding RNAs (lncRNAs) are known as a group of transcripts with over two hundred nucleotides, which lack of or possess a limited capacity to encode proteins [4]. Numerous researches have argued that lncRNAs participate in various biological events, including transcriptional regulation and tumor occurrence [4, 5]. Recent studies also indicated that dysregulated lncRNAs are linked to human tumor development [5]. lncRNA AFAP1-AS1 is a newly discovered tumor-associated lncRNA originated from the antisense strand of the AFAP1 gene [6]. It was reported to be related with multiple malignant tumors, including esophageal cancer, nasopharyngeal cancer (NPC), and tongue squamous cell carcinoma (TSCC) [7–9]. lncRNA AFAP1-AS1 may elevate the protein level of VEGF-C and artemin to enhance esophageal cancer cell invasion and migration. In NPC and TSCC, elevated lncRNA AFAP1-AS1 was found to be related to metastasis and poor prognosis; moreover, lncRNA AFAP1-AS1 silencing could repress NPC and TSCC cell migration and invasion [9, 10]. Nevertheless, the role of lncRNA AFAP1-AS1 in LC remains undetermined.

The article "The Expression of the Long Noncoding RNA AFAP1-AS1 in Laryngeal Carcinoma Affects the Proliferation, Invasion, Migration, and Apoptosis of TU212 Cell Line" was retracted in 2023. Reasons: unreliable results or conclusions; lack of ethics approval or compliance; concerns about the data; concerns about the peer review.

Herein, we aimed to study whether lncRNA AFAP1-AS1 plays a role in the regulation of LC cell proliferation, apoptosis, migration, and invasion. Our results indicated that lncRNA AFAP1-AS1 was elevated in LC. Moreover, loss-of-function assays suggested that lncRNA AFAP1-AS1 acts as an oncogene of LC. Our findings suggested that lncRNA AFAP1-AS1 might act as a potential diagnostic biomarker and therapeutic target for LC.

## 2. Methods

### 2.1. Human Tissues

Twenty-nine LC patients who received therapy between June 2020 and December 2020 at the Otorhinolaryngology Department of the Second Affiliated Hospital of Nanchang University, Jiangxi, China, were included in the study. This population is consisted of 29 males, aged 42-81 (median age = 64.5). Patients did not undergo chemo- or radiotherapy, did not have other tumors, immune system diseases, and blood system diseases, and did not have advanced cardiac, liver, kidney, and other organ dysfunction. The adjacent normal tissues were collected from the 29 LC patients, approximately 1-2 cm away from the tumors as the control group. Informed consents were obtained from all 29 LC patients. Tissues were kept under -80°C until use. The clinicopathologic characteristics of the 29 LC patients are presented in Table 1.

### 2.2. Cell Culture

TU-212 cell line purchased from Beina Bio (BNCC340714) was maintained in DMEM medium plus penicillin/streptomycin and fetal bovine serum (10%). Cells were placed in a humidified condition with 5% CO_2_ at 37°C.

### 2.3. Vector Establishment and Cell Transfection

Add 1 mL of 0.25% trypsin for digestion for 2-3 min, then add 2 mL of complete medium to terminate the digestion, centrifuge at 1,000 r/min for 5 min, remove supernatant and collect the pelleted cells, and resuspend in complete culture medium. After the cell suspension is passaged or inoculated according to the required ratio, take logarithmic growth of cells and placed in 6-well plates and cultured for 24 h, and then, Lipofectamine™ 3000 Kit (Invitrogen, L3000015) was employed to conduct cell transfection. Incubate cells at 37°C for 2-4 days.

The article "The Expression of the Long Noncoding RNA AFAP1-AS1 in Laryngeal Carcinoma Affects the Proliferation, Invasion, Migration, and Apoptosis of TU212 Cell Line" was retracted in 2023. Reasons: unreliable results or conclusions; lack of ethics approval or compliance; concerns about the data; concerns about the peer review.

### 2.4. Quantitative Real-Time PCR Analysis

Total RNAs of LC tissues and cells were extracted using TRIzol reagent (Invitrogen, USA) following the manufacturer's guidance. Then, RNA was reverse transcribed into cDNA using the iScript™ cDNA Synthesis Kit (Bio-Rad, USA). Real-time PCR reaction was conducted on an ABI 7500 system using SYBR Premix Dimer Eraser (Takara, Dalian, China). Sequences of primers are shown in Table 2.

### 2.5. CCK-8 Assay

Briefly, 0.8 × 10^5^ cells/mL were seeded into 96-well plates and CCK-8 reagent was added into each well and allowed for another 2 h of incubation. Absorbance of each well was determined at 450 nm by a Quant Reader (BioTek Instruments, USA). Each sample had three replicates.

### 2.6. Clone Formation Assay

Around 400 cells were placed into 6-well plates and allowed for 14 days of incubation, and culture medium was replaced every two days. Afterwards, colonies were washed by PBS for three times and subjected for crystal violet staining. Colonies with more than fifty cells were counted manually.

### 2.7. EdU Cell Staining

Treated cells were seeded in a 6-well culture plate with three replicates. EdU cell proliferation staining was performed using an EdU kit. For the EdU staining assay, the Cell-Light™ EdU Cell Proliferation Detection Kit (RiboBio) was used. Finally, use Click-iT Additive Solution EdU detected.

### 2.8. Transwell Assay

TU212 cells (2.5 × 10^5^ cell/mL) were included into the top Transwell chamber, and bottom Transwell chamber was filled by FBS-included culture medium. After 24 h of incubation, cells which invade to the lower surface were fixed in methanol and subjected for crystal violet (0.5%) staining.

### 2.9. Wound Healing Assay

Cells seeded in 6-well plate were allowed culturing until full confluence. Then, a scratch was made on the surface of cell layer by a pipette tip followed by PBS washing to discard debris. The scratch was photographed at 0 and 24 h of scratching, and the width was measured.

### 2.10. Flow Cytometry

An apoptosis analysis kit (KeyGEN, KGA1015-1018) was used in flow cytometry analysis. After overnight of fixation with 70% ethanol, cells were subjected for propidium iodide (25 *μ*g/mL) staining for 1 h. Afterwards, a FACSCalibur flow cytometer (Becton Dickinson, USA) was adopted to perform apoptosis analysis.

The article "The Expression of the Long Noncoding RNA AFAP1-AS1 in Laryngeal Carcinoma Affects the Proliferation, Invasion, Migration, and Apoptosis of TU212 Cell Line" was retracted in 2023. Reasons: unreliable results or conclusions; lack of ethics approval or compliance; concerns about the data; concerns about the peer review.

### 2.11. Statistical Analysis

Data analyzed in IBM SPSS21.0 and GraphPad Prism were presented as the mean ± SD. Student's *t*-test or one-way ANOVA was employed to compare difference between groups. A *P* value less than 0.05 was considered statistically significant.

## 3. Results

### 3.1. lncRNA AFAP1-AS1 Was Elevated in LC

We firstly tested lncRNA AFAP1-AS1 expression in normal control (NC, *n* = 29) and LC (*n* = 29) tissues using qRT-PCR. Result indicated a remarkable elevation of lncRNA AFAP1-AS1 in LC (Figure 1). Association between lncRNA AFAP1-AS1 level and LC patients' clinicopathologic characteristics was also investigated. LC patients were divided into the low (*n* = 8) and high (*n* = 21) lncRNA AFAP1-AS1 groups. As expected, elevated lncRNA AFAP1-AS1 expression was linked to T-classification, TNM stage, and tumor differentiation, but irrelevant to other factors, including age and gender (Table 1).

### 3.2. lncRNA AFAP1-AS1 Was Successfully Silenced in TU212 Cells

To study lncRNA AFAP1-AS1 function in TC, three specific shRNAs target lncRNA AFAP1-AS1 (sh#1, sh#2, and sh#3) were designed and transfected into TU212 cells. Green fluorescence was observed in the sh-NC and sh-RNAs transfected groups, suggesting that sh-AFAP1-AS1s and sh-NC were successfully transfected into TU212 cells (Figure 2). As shown by qRT-PCR results, relative lncRNA AFAP1-AS1 expression in TU212 cells was dramatically decreased by three shRNAs compared to the mock group (Figure 3).

### 3.3. lncRNA AFAP1-AS1 Silencing Repressed TU212 Cell Proliferation

Afterwards, the influences of lncRNA AFAP1-AS1 silencing on TU212 cell proliferation viability were tested. A remarkable viability repression was observed in CCK-8 assay in the lncRNA AFAP1-AS1 silenced group (Figure 4). And, we showed that the number of colonies formed by lncRNA AFAP1-AS1 silenced cells was dramatically reduced (Figure 5). The repressive effects of lncRNA AFAP1-AS1 silencing on TU212 cell proliferation viability were further supported by the results from EdU staining (Figure 6).

### 3.4. lncRNA AFAP1-AS1 Silencing Repressed TU212 Cell Migration and Invasion

Impacts of lncRNA AFAP1-AS1 silencing on LC migration and invasion were also tested *in vitro*. By using Transwell chambers coated with Matrigel, we demonstrated that lncRNA AFAP1-AS1 silencing led to a remarkable repressive effect on TU212 cell invasion (Figure 7). Additionally, in wound healing assay, a significant repression of migratory capacity was observed in lncRNA AFAP1-AS1 silenced TU212 cells (Figure 8).

### 3.5. lncRNA AFAP1-AS1 Silencing Facilitated TU212 Cell Apoptosis

Finally, the impacts of lncRNA AFAP1-AS1 silencing on LC cell apoptosis were estimated via flow cytometry, as results indicated that the apoptosis rate was significantly higher in the lncRNA AFAP1-AS1 silenced group compared to the mock and sh-NC groups (Figure 9).

The article "The Expression of the Long Noncoding RNA AFAP1-AS1 in Laryngeal Carcinoma Affects the Proliferation, Invasion, Migration, and Apoptosis of TU212 Cell Line" was retracted in 2023. Reasons: unreliable results or conclusions; lack of ethics approval or compliance; concerns about the data; concerns about the peer review.

## 4. Discussion

The etiology of LC is poorly identified so far [11]. Epidemiological data confirms that it is related to factors including smoking and drinking, viral infection, environmental and occupational factors, radiation, lack of trace elements, and sexual hormone metabolism disorders [12]. At present, the clinical treatment of laryngeal cancer mainly adopts multidisciplinary comprehensive treatment with surgery as the mainstay [12, 13]. Currently, it has been well recognized that the ideal goals of the management of laryngeal cancer are to completely eradicate tumor lesions while preserving and reconstructing the function of the larynx as much as possible and to improve the patient's quality of life [13]. Therefore, it is particularly important to explore the mechanism of LC tumorigenesis from the molecular level.

Recently, dysregulated expression or functions of lncRNAs have been reported in almost all kinds of tumors, and evidence also suggested an involvement of lncRNAs in all steps of tumor occurrence and progression [4, 14]. lncRNAs are widely believed to exert critical impacts on diagnosis, management, and prognosis of tumors [4, 15]. The discovery of lncRNA provides a novel direction for studying gene regulation. It can act as a carcinogenic or tumor repressive factor to participate in tumor proliferation, invasion, migration, and apoptosis [4, 16]. Numerous lncRNAs have been found to be elevated or downregulated in LC, and evidence also demonstrated that lncRNAs play an important role in regulating LC cell growth, apoptosis, invasion, and migration through various of mechanisms [17–19]. lncRNA AFAP1-AS1 has been revealed to play a role in numerous cancers by a large of studies. For instance, it was reported to be an oncogene in gastric cancer by regulating FGF7 expression via miR-155-5p [20]. lncRNA AFAP1-AS1 also promotes the occurrence and development of osteosarcoma by competitively binding miR-497 [21]. lncRNA AFAP1-AS1 is also elevated in lung cancer and mediates lung cancer cell inhibition by modulating the expression of miR-545-3p [22]. However, there are few studies focusing on the role of lncRNA AFAP1-AS1 in LC. Only Yuan et al. have shown that lncRNA AFAP1-AS1 increases RBPJ expression through negative regulation of miR-320a, and the overexpression of RBPJ rescues the repressive effects of lncRNA AFAP1-AS1 on LC [23]. Thus, it is reasonable to believe that AFAP1-AS1 holds a carcinogen potential to participate in the process of tumors. Yet, the specific mechanism of occurrence and development needs to be further studied.

The article "The Expression of the Long Noncoding RNA AFAP1-AS1 in Laryngeal Carcinoma Affects the Proliferation, Invasion, Migration, and Apoptosis of TU212 Cell Line" was retracted in 2023. Reasons: unreliable results or conclusions; lack of ethics approval or compliance; concerns about the data; concerns about the peer review.

Herein, we tested the expression of lncRNA AFAP1-AS1 in LC tissues and cells, and we also studied its role in LC *in vitro* using TU212 cells. lncRNA AFAP1-AS1 was reported to be an oncogene of a variety of cancers. Similarly, our results also suggested that lncRNA AFAP1-AS1 promotes LC progression *in vitro*.

Although the data from our study revealed that AFAP1-AS1 is an oncogene of LC, there are still a few limitations. First, sample size of the study is not large enough, but we believe that it has sufficient statistical power. Second, we did not explore the mechanism of lncRNA AFAP1-AS1 in LC.

## 5. Conclusions

lncRNA AFAP1-AS1 is highly presented in LC and is related to the clinicopathological characteristics of LC patients. Moreover, *in vitro* loss-of-function assays suggested that lncRNA AFAP1-AS1 acts as an oncogene of LC.

## Figures and Tables

**Figure 1:** Relative lncRNA AFAP1-AS1 level in NC and LC tissue samples. lncRNA AFAP1-AS1 was sharply elevated in the LC group. ^∗^*P* < 0.05.

**Figure 2:** Confocal images showing that sh-AFAP1-AS1 and sh-NC were successfully transfected into TU212 cells. Green fluorescence was observed in the sh-NC and sh-RNAs transfected groups.

**Figure 3:** Knockdown efficiency of three shRNAs target AFAP1-AS1 (sh#1, sh#2, and sh#3) were tested by qRT-PCR in TU212 cells. All three shRNAs dramatically decreased lncRNA AFAP1-AS1 level. ^∗∗^*P* < 0.01.

**Figure 4:** Impacts of lncRNA AFAP1-AS1 silencing on TU212 cell viability were estimated via CCK-8 kit. lncRNA AFAP1-AS1 silencing repressed TU212 cell viability. ^∗∗∗^*P* < 0.001.

**Figure 5:** Impacts of AFAP1-AS1 silencing on TU212 cell clonogenicity were tested by colony formation assay. (a) Representative images showing the colonies formed by treated TU212 cells. (b) Statistical analysis of clone number in each group.

**Figure 6:** EdU staining results showing the influences of AFAP1-AS1 silencing on TU212 cell proliferation. (a) Representative images showing the EdU-stained TU212 cells. (b) Statistical analysis of EdU staining.

**Figure 7:** Invasive capacity of TU212 cell was assessed through Transwell chamber with Matrigel after transfection with si-AFAP1-AS1 or si-NC. (a) Representative images showing the invasive cells in each group. (b) Statistical analysis of the number of invasive cells.

**Figure 8:** Migratory capacity of TU212 cell was assessed via wound healing assay after transfection with si-AFAP1-AS1 or si-NC. (a) Representative images showing the wound width. (b) Statistical analysis of the width of wound from each group.

The article "The Expression of the Long Noncoding RNA AFAP1-AS1 in Laryngeal Carcinoma Affects the Proliferation, Invasion, Migration, and Apoptosis of TU212 Cell Line" was retracted in 2023. Reasons: unreliable results or conclusions; lack of ethics approval or compliance; concerns about the data; concerns about the peer review.

**Figure 9:** Flow cytometry analysis results showing the impacts of transfection with si-AFAP1-AS1 or si-NC on TU212 cell apoptosis. (a) Representative images showing the flow cytometry analysis of cells. (b) Statistical analysis of apoptosis rate.

**Table 1:** Relationship between lncRNA AFAP1-AS1 expression and clinicopathological features in patients with LC.

Parameter	Total (*n* = 29)	lncRNA AFAP1-AS1		*χ* ^2^	*P*
		Low (*n* = 8)	High (*n* = 21)		
Age (years)					
<60	5	3 (60.0%)	2 (40.0%)	3.178	0.075
≥60	24	5 (20.8%)	19 (79.2%)		
Gender					
Female	29	8 (27.6%)	21 (72.4%)	—	0.999
Male	0	0	0		
T-classification					
T1-T2	10	6 (60.0%)	4 (40.0%)	8.028	0.004^∗∗^
T3-T4	19				
(TNM)		2 (10.5%)	17 (89.5%)		
I-II	8			6.741	0.009^∗∗^
III-IV	21	5 (62.5%)	3 (37.5%)		
Tumor differentiation		3 (14.3%)	18 (85.7%)		
Well/moderate	23	4 (17.4%)	19 (82.6%)	5.784	0.016^∗^
Poor	6	4 (66.7%)	2 (33.3%)		

^∗^ *P* < 0.05 and ^∗∗^*P* < 0.05.

**Table 2:** Sequences of primers.

Gene symbols	Sequences
GAPDH	F: ATGGGGAAGGTGAAGGTCG
	R: TCGGGGTCATTGATGGCAACAATA
Primer of AFAP1-AS1	F: ATAAGAATGGCTTGCTGTGGAC
	R: GGTTGGTGCGGTTGGAATAG
AFAP1-AS1-siRNA1	F: GATCCGCACGGAGTGTGGCACAATAACTCGAGTTATTGTGCCACACTCCGTGCTTTTTGC
	R: GGCCGCAAAAAGCACGGAGTGTGGCACAATAACTCGAGTTATTGTGCCACACTCCGTGCG
AFAP1-AS1-siRNA2	F: GATCCGCACGGAGTGTGGCACAATAACTCGAGTTATTGTGCCACACTCCGTGCTTTTTGC
	R: GGCCGCAAAAAGCACGGAGTGTGGCACAATAACTCGAGTTATTGTGCCACACTCCGTGCG
AFAP1-AS1-siRNA3	F: GATCCGCACGGAGTGTGGCACAATAACTCGAGTTATTGTGCCACACTCCGTGCTTTTTGC
	R: GGCCGCAAAAAGCACGGAGTGTGGCACAATAACTCGAGTTATTGTGCCACACTCCGTGCG
si-NC	F: TAGTTATTAATAGTAATCAATTACGGGGTCATTAGTTCATAGCCCATATATGGAGT
	R: GTTCTTTCCTGCGTTATCCCCTGATTCTGTGGATAACCGTATTACCGCCATGCAT

## Data Availability

The datasets used and analysed during this study are available from the corresponding author on reasonable request.
